The article "Effect of Bairui Granule on Inflammatory Mediators in Induced Sputum, Leukotriene C4, and EOS in Peripheral Blood of Children with Cough Variant Asthma" was retracted in 2023. Reasons: signs of a paper mill; suspected computer-generated content; unreliable results or conclusions; concerns about the data.

# Effect of Bairui Granule on Inflammatory Mediators in Induced Sputum, Leukotriene C4, and EOS in Peripheral Blood of Children with Cough Variant Asthma

**DOI:** 10.1155/2022/2657994

**Published:** 2022-06-08

**Authors:** Yi Shen, Min Lu, Qiuyan Xu, Lu Liu, Zhi Cheng

**Affiliations:** Department of Paediatrics, The Affiliated Suzhou Science &Technology Town Hospital of Nanjing Medical University, China

## Abstract

**Objective:**

To study the effect of Hanchuan Zupa granule combined with conventional western medicine in the treatment of children with bronchial asthma.

**Methods:**

98 cases in Fengrun District People's Hospital of Tangshan City from June 2018 to February 2021 were selected. The control group was given oxygen therapy, antibiotics, and aerosol inhalation of quick acting *β* 2 receptor agonist, glucocorticoid, and other conventional western medicine treatment, while the observation group was treated with Bairui granule on the basis of the control group. The course of treatment of the two groups was 1 week.

**Results:**

After treatment, the levels of sputum IL-4, IL-17, neu, and ECP in the two groups decreased, and the observation group was lower than the control group (*P* < 0.05). The levels of EOS, CXCR4, LTB4, and SDF-1 in peripheral blood of the two groups were lower than those in the control group (*P* < 0.05). The daytime cough, night cough, and TCM syndrome scores of the two groups were decreased, and the observation group was lower than the control group (*P* < 0.05).

**Conclusion:**

Bairui granule combined with conventional western medicine in the treatment of children with bronchial asthma, the curative effect is worthy of affirmation, can effectively improve cough symptoms, reduce EOS, CXCR, LTB4, SDF-1 levels, inhibit airway inflammation, and has good clinical application value.

## 1. Introduction

Bronchial asthma (abbreviated as asthma) mainly manifests as wheezing, coughing and chest tightness, shortness of breath, and other symptoms. Exercise and infection and other triggers immediately occur when affected and other characteristics [1]. At present, the prevalence of childhood asthma in my country is not optimistic. According to data, the prevalence of children under the age of 14 in Chinese cities has been increasing year by year from 1990 to 2010, reaching more than 3.02% [2]. There are various factors affecting the onset of asthma, which are not only related to individual factors such as physical fitness, race, genetics, etc. but also researches believe that environmental factors such as air pollution and global climate abnormalities are the main causes of asthma [3]. Since the pathogenesis of asthma has not been clarified, and there is no clinical cure, management and control are mainly based on the symptoms of children to avoid overtreatment or undertreatment. The guidelines recommend long-term medication regimens with long-acting *β*2 receptor agonists and inhaled glucocorticoids. Hormones are the main factors [4], but these programs still have many risks, such as easy relapse after stopping the drug, and drug resistance after long-term use. In this study, the use of Bairui granules combined with western medicine to treat children with asthma in hospitals was compared with those treated with western medicine alone, and satisfactory results were obtained.

The article "Effect of Bairui Granule on Inflammatory Mediators in Induced Sputum, Leukotriene C4, and EOS in Peripheral Blood of Children with Cough Variant Asthma" was retracted in 2023. Reasons: signs of a paper mill; suspected computer-generated content; unreliable results or conclusions; concerns about the data.

## 2. Materials and Methods

### 2.1. General Information

A total of 98 children with acute exacerbation of asthma who were treated in the outpatient and inpatient from June 2018 to February 2021 were selected as the study objects, including 58 males and 40 females, aged 6-12 years old. The average age is (8.96 ± 1.03) years old. The screening process for included patients is shown in Figure 1. Using the random number table method, 98 children were included in the control group and the observation group according to the order of visits. There were 49 patients in the control group, including 28 males and 21 females, aged 6-12 years, with an average of (9.15 ± 1.06) years, and the course of asthma was 3 months to 4 years, with an average of (1.59 ± 0.33) years, and the acute phase was 2 years. ~2 days, average (12.32 ± 2.24) h, 49 cases in the severe control group, 28 males and 21 females, aged 6-12 years, mean (9.15 ± 1.06) years old, asthma duration 3 months to 4 years, mean (1.59 ± 0.33) years, acute phase 2 ~ 2 d, average (12.32 ± 2.24) h; among them, there were 15 patients with mild asthma and 34 patients with moderate asthma. There were 49 patients in the observation group, including 30 males and 19 females, aged 6 to 12 years, with an average of (9.20 ± 1.05) years old, the course of asthma was 3 months to 5 years, with an average of (1.64 ± 0.35) years, and the acute phase was 3 hours. ~3 d, with an average of (12.20 ± 2.36) h, among which, 18 patients with mild asthma and 31 patients with moderate asthma. Comparing the general information of the two groups of children, the difference was not statistically significant (*P* > 0.05), and it was comparable (Table 1). This study was reviewed and approved by the ethics committee.

### 2.2. Diagnostic Criteria

According to the Guidelines for the Diagnosis and Prevention of Bronchial Asthma in Children (2016 Edition) [5], the diagnostic criteria, staging, and grading criteria for asthma are formulated: (1) asthma: ① with repeated wheezing, shortness of breath, coughing, and other manifestations, often in attacks at night and early in the morning are related to factors such as cold air, allergens, and mood swings; ② expiration is prolonged, the lungs can be heard and mainly expiratory wheezing; ③ It can be relieved after antiasthma treatment; ④ exclude the symptoms and signs caused by other diseases; ⑤ examination found that there is reversible airflow limitation, the bronchial provocation test is positive, and the intraday variation rate of the maximum peak expiratory flow within 2 consecutive weeks exceeds 13%. (2) The stage is the acute attack stage: the sudden onset of asthma symptoms or the sudden onset of the original symptoms aggravate. (3) grading: ① mild: shortness of breath can occur during activities, continuous speaking, can be lying flat, accompanied by slight anxiety, can be heard and scattered wheezing; ② moderate: shortness of breath can occur when speaking, speaking cannot continue, like sitting, accompanied by anxiety, irritability, three-concave signs, loud wheezing, increased heart rate, and respiratory frequency; ③ severe: shortness of breath can occur when resting, words can be spoken, anxiety is serious, and forward. In the arch position, diffuse, biphasic, and loud wheezing can be heard in both lungs, blood oxygen saturation is lower than 90%, and heart rate and respiratory rate are significantly increased.

The article "Effect of Bairui Granule on Inflammatory Mediators in Induced Sputum, Leukotriene C4, and EOS in Peripheral Blood of Children with Cough Variant Asthma" was retracted in 2023. Reasons: signs of a paper mill; suspected computer-generated content; unreliable results or conclusions; concerns about the data.

According to the Consensus of Traditional Chinese Medicine Diagnosis and Treatment of Bronchial Asthma (2012) [J] [6], the TCM dialectical standard for cold asthma during asthma attack is established: (1) main symptoms: shortness of breath, wheezing in the throat, wheezing, and holding breath inverse; (2) secondary syndrome and tongue and pulse conditions: low cough, fullness and congestion in the chest, less white phlegm, prefers hot drinks, cold limbs and fear of cold, dull complexion, white tongue and slippery coating, and tight pulse string; in line with the main syndrome and two secondary syndromes can be diagnosed as cold asthma syndrome.

### 2.3. Inclusion Criteria

(1) Meet the diagnostic criteria of asthma; (2) meet the TCM syndrome differentiation criteria of “cold asthma syndrome;” (3) in the acute attack stage; (4) the condition is mild to moderate; (5) age 6-12 between the ages of; (6) no other treatment measures were taken before the consultation, and other clinical studies were not taken; (7) the guardian of the child was aware of the contents of this study and signed an informed consent form voluntarily.

### 2.4. Exclusion Criteria

(1) A history of drug allergy; (2) combined with other respiratory diseases such as bronchiectasis; (3) combined with severe heart, liver, and kidney diseases, and congenital diseases; (4) intolerance to hormones; (5) combined Immune system diseases; (6) poor lung function, unable to persist in completing this study; (7) poor compliance, unable to complete the treatment.

The article "Effect of Bairui Granule on Inflammatory Mediators in Induced Sputum, Leukotriene C4, and EOS in Peripheral Blood of Children with Cough Variant Asthma" was retracted in 2023. Reasons: signs of a paper mill; suspected computer-generated content; unreliable results or conclusions; concerns about the data.

### 2.5. Method

The control group received conventional Western medical treatment during the acute attack of asthma, including oxygen therapy (to maintain blood oxygen saturation above 94%), antibacterial drug application, aerosol inhalation of fast-acting *β*2 receptor agonists (salbutamol, terbutaline, etc.), and sugar corticosteroid application (aerosol inhalation of budesonide or oral prednisone or intravenous injection of methylprednisolone). The observation group was added with Bairui granules (Anhui Jiuhua Huayuan Pharmaceutical Co., Ltd., National Medicine Standard Z20090694, specification 5 g) on the basis of the control group, 6 g/time, 3 times/day for one week.

### 2.6. Observation Items

All items were tested before and after the treatment and performed by the same doctor. (1) Detection of induced sputum content: ① collect sputum: at 8 am before and after treatment (without eating), first use a pulmonary function meter to detect the child's forced vital capacity (FEV1) in the first second, and take the average value after three consecutive measurements baseline, then use normal saline to rinse mouth fully, instruct children to inhale 200 *μ*g of salbutamol (2 sprays), and then nebulize hypertonic saline (concentration of 3-5%, adjust hypertonic saline from low to low according to the presence or absence of sputum) (high inhalation) for 20 minutes, encourage the child to cough up deep sputum, and collect the sputum into a 50 mL sterile bottle. During this process, closely observe the performance of the child. If symptoms such as dyspnea, wheezing, cough, etc. occur, or the FEV1 predicted value is low, immediately stop at 60%, and take corresponding emergency measures; ② sputum treatment: first weigh the sputum, add 2 times the weight of 0.1% dithiothreitol, 37% water bath for 30 minutes, shake well, and then centrifuge (1000 r/min, 15 min), take the supernatant, make cell smears, wright stain, count 400 nonsquamous epithelial cells under light microscope, observe neutrophils (NEU), and eosinophils (ECP) percentage. The detection kit was purchased from R&D Company in the United States.

(2) Detection of blood indicators: take 5 mL of fasting cubital venous blood before and after treatment in children, and calculate the EOS count in peripheral blood under light microscope; use flow cytometry to detect the expression level of chemokine receptor 4 (CXCR4) in peripheral blood of children. The serum was separated and stored at low temperature were detected by ELISA. The detection kit was purchased from R&D Company in the United States.

(3) Symptom evaluation: ① clinical symptom score: score the day and night cough of the child before and after treatment, and score 0, 1, 2, and 3 according to no, mild, moderate, and severe. The higher the score, the higher the score. The more severe the cough. ② Traditional Chinese medicine syndrome: score the primary and secondary symptoms of the child before and after treatment, and divide them into four levels: none, mild, moderate, and severe.

(4) Adverse reactions: observe the adverse reactions during medication.

The article "Effect of Bairui Granule on Inflammatory Mediators in Induced Sputum, Leukotriene C4, and EOS in Peripheral Blood of Children with Cough Variant Asthma" was retracted in 2023. Reasons: signs of a paper mill; suspected computer-generated content; unreliable results or conclusions; concerns about the data.

### 2.7. Efficacy Criteria

The efficacy evaluation criteria were formulated: ① clinical control: the children's cough symptoms disappeared completely, and the TCM syndrome scores were reduced by more than 95%; ② significantly effective: the child's cough symptoms are significantly improved; ③ effective: the child's cough symptoms are alleviated, and the TCM syndrome score is reduced by more than 30%; ④ ineffective: the child has no cough symptoms. Significant changes, even worsening, the reduction of TCM syndrome scores is less than 30%. Total effective rate = (clinical control in this group + markedly effective + effective)/number of cases in the group × 100%.

### 2.8. Statistical Methods

SPSS21.0 software was used for data analysis, measurement data were expressed as mean ± standard deviation (±*S*), two-sample independent *t* test was used for comparison between groups, and the difference was considered statistically significant when *P* < 0.05.

## 3. Results

### 3.1. Comparison of IL-4, IL-17, NEU, and ECP Levels in Sputum

After treatment, the levels of IL-4, IL-17, NEU, and ECP in the sputum of the two groups decreased. And the observation group is lower than the control group (*P* < 0.05), see Table 2.

### 3.2. Comparison of Peripheral Blood EOS, CXCR4, and Serum LTB4 and SDF-1 Levels after and before Therapy between the Two Groups

After treatment, the levels of EOS, CXCR4, and serum LTB4 and SDF-1 in the two groups were decreased, and observation, the group is lower than the control group (*P* < 0.05), see Table 3.

### 3.3. Comparison of Scores of Cough Symptoms and TCM Syndrome Scores between the Two Groups after and before Therapy

After treatment, the scores of day cough, night cough, and TCM syndromes were lower in the two groups, and the observation group was lower than control group (*P* < 0.05), see Table 4.

### 3.4. Comparison of the Efficacy of the Two Groups

Compared with the control group, the total effective rate of the observation group was higher, and the difference was statistically significant (*P* < 0.05), see Table 5.

The article "Effect of Bairui Granule on Inflammatory Mediators in Induced Sputum, Leukotriene C4, and EOS in Peripheral Blood of Children with Cough Variant Asthma" was retracted in 2023. Reasons: signs of a paper mill; suspected computer-generated content; unreliable results or conclusions; concerns about the data.

### 3.5. Comparison of Adverse Reactions between the Two Groups

No serious adverse reactions occurred in the two groups, and 2 gastrointestinal reactions occurred in the observation group, which recovered spontaneously without treatment.

## 4. Discussion

Asthma is characterized by airway allergic inflammation, airway hyperresponsiveness, and airway remodeling, in which inflammation is the central link and hyperresponsiveness is the essence [7–9]. The pathogenesis of asthma is complicated, and the current mainstream theories generally study it from the aspects of airway inflammation mechanism, genetic mechanism, immune, and allergic reaction mechanism [8, 10–12]. The mechanism of airway inflammation is studied from the three aspects of inflammatory cells (ECP, NEU, lymphocytes, etc.), inflammatory mediators (LTB4), and cytokines (IL-4, IL-17, etc.) from the chronic inflammatory response of asthma [13].

The etiology of asthma is complex and is generally considered to be the result of the interaction of a variety of pathogenic factors, but it is also about internal and external causes. It is caused by the unfavorable body fluid infusion and accumulation in the lungs to form “sputum phlegm” [14], which is mostly caused by the dysfunction of the spleen, lungs, and kidneys; or due to insufficient congenital endowment, phlegm, and drinking endogenously; or due to excessive eating and spicy; fatness, coldness, and injury to the spleen and stomach, loss of movement of the spleen, obstruction of phlegm and blood stasis, and upset of the lung; or due to cold pathogens invading the lungs, the lungs fail to declare and subdue, and cold phlegm is endogenous [15–18]. The external causes are sudden changes in climate, eating disorders, emotional disorders, overwork, and other stimuli to the body, which can induce “phlegm” [19–22]. The main pathogenesis is wind and cold attacking the lungs. The treatment principle is to warm the lungs to resolve phlegm, relieve cough, and relieve asthma.. The main extract of Bairui granules is thyme grass. The history is recorded in the “Book of Sketches.” It is a perennial parasitic herb [23]. The kaempferol contained in thyme grass has anticough and antiepidemic effects; thyme, kaempferol, and its 3-glucorhamnoside and succinic acid have broad-spectrum antibacterial activity in vitro; D-mannitol, succinic acid has an antiasthmatic effect [24]; at the same time, pyramid particles can prevent virus replication by binding viral nucleic acid or capsid protein. It is considered to be a broad-spectrum antibacterial and anti-inflammatory drug. Its efficacy can reduce the frequency of coughing and improve the trachea. The ability to expectoration of sputum is thereby improving the patient's lung function [25].

The article "Effect of Bairui Granule on Inflammatory Mediators in Induced Sputum, Leukotriene C4, and EOS in Peripheral Blood of Children with Cough Variant Asthma" was retracted in 2023. Reasons: signs of a paper mill; suspected computer-generated content; unreliable results or conclusions; concerns about the data.

The scores of cough symptoms and TCM syndrome scores were lower than those of the control group (*P* < 0.05), confirming that Bairui granules have a good therapeutic effect on asthma. It can effectively improve the symptoms of cough, relieve the symptoms of traditional Chinese medicine, and has a definite clinical effect. IL-4 is a marker of inflammatory cells that can mediate airway inflammation, airway remodeling, and airway hyperresponsiveness, and its level is positively correlated with the severity of the disease [26]. IL-17 is an important member of asthma-related factors. By inducing epithelial cells, endothelial cells, and fibroblasts to secrete a variety of inflammatory factors, increasing the expression of intercellular adhesion factor 1 [27], it is widely involved in the occurrence and development of asthma. Chronic airway inflammation in asthma is mainly manifested as infiltration of inflammatory cells such as ECP, ENU, and lymphocytes. ECP is the active secretion product of eosinophils, and together with eosinophils, it induces the activation of nuclear factor (NF-*κ*B), initiates the expression of inflammation-related genes, and stimulates and amplifies the inflammatory response [28]. EOS is an inflammatory effector cell in the pathogenesis of asthma. It can release and synthesize a variety of inflammatory cytokines; induce or aggravate allergic reactions; damage epithelial, mucosa, smooth muscle, and other tissues; and participate in asthma by producing leukotrienes and toxic granule proteins. LTB4 is a chemokine produced by activated mononuclear macrophages and NEU. It has an effect on the aggregation and activation of NEU and ECP after the action of antigen. At the same time, it has a strong bronchoconstriction effect, which can shrink the trachea and increase the resistance in the airway. Reduce lung function [29]. SDF-1 can bind to CXCR4 on a variety of cells. The activated SDF-1/CXCR4 pathway can chemoattract inflammatory cells. Animal experiments have confirmed that the levels of SDF-1 and CXCR4 in asthmatic rats are higher than those in the control group [30–32].

In summary, the use of Bairui granules combined with conventional Western medicine to treat children with bronchial asthma is worthy of affirmation. It can effectively improve cough symptoms; reduce EOS, CXCR, LTB4, and SDF-1 levels; and inhibit airway inflammation. It has good clinical applications. However, the study also has shortcomings, the observation time is short, and the long-term follow-up of children cannot be followed to evaluate the long-term efficacy.

The article "Effect of Bairui Granule on Inflammatory Mediators in Induced Sputum, Leukotriene C4, and EOS in Peripheral Blood of Children with Cough Variant Asthma" was retracted in 2023. Reasons: signs of a paper mill; suspected computer-generated content; unreliable results or conclusions; concerns about the data.

## Figures and Tables

**Figure 1:** Screening process for included patients.

**Table 1:** Comparing the general information of the two groups of children ($\bar{x}\pm s,n$).

Group	Males/females	Age (years)	Asthma course (years)	Acute course (*h*)	Severity (mild/moderate)
Control group (*n* = 49)	28/21	9.15 ± 1.06	1.59 ± 0.33	12.32 ± 2.24	15/34
Observation group (*n* = 49)	30/19	9.20 ± 1.05	1.64 ± 0.35	12.20 ± 2.36	18/31
*P*	>0.05	>0.05	>0.05	>0.05	>0.05

**Table 2:** Comparison of IL-4, IL-17, NEU, and ECP levels in sputum before and after treatment between the two groups ().

Group	IL-4 (ng/L)		IL-17 (ng/L)		NEU (%)		ECP (%)	
	Before therapy	After treatment	Before therapy	After treatment	Before therapy	After treatment	Before therapy	After treatment
Control group (*n* = 49)	24.36 ± 4.53	15.48 ± 3.86^∗^	457.28 ± 36.85	315.54 ± 30.38^∗^	31.58 ± 5.26	28.16 ± 4.43^∗^	10.96 ± 2.71	2.83 ± 0.64^∗^
Observation group (*n* = 49)	25.01 ± 4.75	12.54 ± 2.85^∗^	465.72 ± 38.55	278.16 ± 31.39^∗^	32.03 ± 5.48	26.35 ± 4.18^∗^	11.25 ± 2.56	1.95 ± 0.49^∗^
*t*	0.693	4.289	1.108	5.990	0.415	2.080	0.545	7.642
*P*	0.245	0.000	0.135	0.000	0.340	0.020	0.294	0.000

Note: compared with before therapy in the same group, ∗*P* < 0.05.

**Table 3:** Comparison of peripheral blood EOS, CXCR4, and serum LTB4 and SDF-1 levels after before therapy between the two groups ($\bar{x}\pm s$).

Group	EOS (N/HP)		CXCR4		LTB4 (ng/L)		SDF-1 (ng/L)	
	Before therapy	After treatment	Before therapy	After treatment	Before therapy	After treatment	Before therapy	After treatment
Control group (*n* = 49)	36.15 ± 2.75	15.37 ± 1.86^∗^	22.86 ± 4.16	7.05 ± 1.12^∗^	175.26 ± 30.51	133.81 ± 22.56^∗^	589.27 ± 83.16	470.14 ± 68.49^∗^
Observation group (*n* = 49)	35.89 ± 3.54	11.06 ± 1.67^∗^	23.38 ± 3.85	5.79 ± 0.84^∗^	180.63 ± 35.42	118.75 ± 25.34^∗^	603.64 ± 79.48	415.74 ± 64.85^∗^
*t*	0.406	12.069	0.642	6.300	0.804	3.107	0.874	4.037
*P*	0.343	0.000	0.261	0.000	0.212	0.001	0.192	0.000

Note: compared with before therapy in the same group, ∗*P* < 0.05.

**Table 4:** Comparison of cough symptom scores and TCM syndrome scores between the two groups after before therapy ($\bar{x}\pm s$).

Group	Day cough		Night cough		TCM syndrome	
	Before therapy	After treatment	Before therapy	After treatment	Before therapy	After treatment
Control group (*n* = 49)	1.35 ± 0.18	0.65 ± 0.10	1.86 ± 0.27	0.97 ± 0.30	11.84 ± 2.18	6.58 ± 1.15
Observation group (*n* = 49)	1.32 ± 0.20	0.48 ± 0.11	1.81 ± 0.30	0.64 ± 0.22	12.28 ± 2.30	5.34 ± 1.27
*t*	0.780	8.005	0.867	6.209	0.972	5.066
*P*	0.219	0.000	0.194	0.000	0.167	0.000

**Table 5:** Comparison of the efficacy of the two groups (*n*).

Group	Number of cases	Clinical control	Markedly effective	Efficient	Invalid	Total effective rate%
Control group	49	21	13	10	5	89.80
Observation group	49	10	15	11	13	73.47
*t*						4.356
*P*						0.037

The article "Effect of Bairui Granule on Inflammatory Mediators in Induced Sputum, Leukotriene C4, and EOS in Peripheral Blood of Children with Cough Variant Asthma" was retracted in 2023. Reasons: signs of a paper mill; suspected computer-generated content; unreliable results or conclusions; concerns about the data.

## Data Availability

No data were used to support this study.
